The article "Evaluation of Sepsis-1 and Sepsis-3 Diagnostic Criteria in Patients with Sepsis in Intensive Care Unit" was published in 2023. Journal: J Healthc Eng.

# Evaluation of Sepsis-1 and Sepsis-3 Diagnostic Criteria in Patients with Sepsis in Intensive Care Unit

**DOI:** 10.1155/2023/3794886

**Published:** 2023-07-07

**Authors:** Qianying Song, Weiyu Fei

**Affiliations:** Department of EICU, The Second Hospital of Dalian Medical University, 467 Zhongshan Road, Shahekou District, Dalian 116023, China

## Abstract

**Background:**

The use of SIRS and SOFA criteria in diagnosing sepsis among patients has been characterized by increasingly growing criticism. Indeed, the definition of sepsis has attracted significant controversy in history across medical and academic realms.

**Methods:**

The study used the Medical Information Mart for Intensive Care-III (MIMIC-III) database in assessing the effectiveness of the SIRS and SOFA diagnostic criteria. It ascertained the severity and specificity of sepsis infection in ICU patients. The Medical Information Mart for Intensive Care-III (MIMIC-III) database was established by the Beth Israel Deaconess Medical Center (BIDMC) and MIT's Computational Physiology Laboratory. The database is a voluminous single-center database containing information pertaining to 38,000 adults who were admitted to the BIDMC in the 11 years leading up to 2012. The identification of patients with sepsis was conducted using the International Classification of Diseases (ICD-10-CM) diagnosis codes.

**Results:**

The analysis of data for this study was based on the chi-square test, which is significant in comparing the specificity, mortality, and sensitivity of the data. The process of screening the MIMIC-III database resulted in the identification of 21,368 patients with infections from the hospital admissions in the database. The results also indicate a significantly higher mortality rate within 28 days of admission in sepsis-3 patients compared with sepsis-1. In this experiment, we limited the study period to 28 days to restrict the potential of mortality caused by other factors. Additionally, we evaluated the clinical factors associated with the sepsis-1 or sepsis-3 and found out similar results in the analysis for sepsis-1 and sepsis-3.

**Conclusions:**

The study results also portray numerous challenges in using the sepsis-3 criteria as a diagnostic tool. In particular, the ICD-10-CM diagnosis approach was limiting because it inhibited the measure of uncertainty of infection present at the beginning of the two diagnostic criteria of sepsis-1 and sepsis-3.

## 1. Introduction

The definition of sepsis has attracted significant controversy in history across medical and academic realms. The first definition (sepsis-1) was adopted in 1992 based on the systematic inflammatory response syndrome (SIRS) [1]. The second definition (sepsis-2) was then proposed in 2001 based on redefined diagnostic criteria of the first definition. The ineffectiveness of these diagnostic criteria gave birth to the third definition (sepsis-3), which eliminated SIRS and severe sepsis concepts [2]. Instead, the third definition identified life-threatening dysfunction arising out of a dysregulated host response to infection as central to the diagnosis of sepsis. It was based on the attainment of a score of 2 or more than 2 of the sequential organ failure assessment (SOFA) score.

The article "Evaluation of Sepsis-1 and Sepsis-3 Diagnostic Criteria in Patients with Sepsis in Intensive Care Unit" was published in 2023. Journal: J Healthc Eng.

The controversy regarding the definition of sepsis is a matter of grave concern across both academic and professional spheres of medical research [3]. In particular, sepsis is identified as a leading contributor to high mortality across the world [4]. Besides, sepsis is also associated with an increasingly growing health burden worldwide, thus threatening public health systems. It is not surprising that sepsis has drawn considerable attention from both researchers and physicians with an attempt to understand its implications on public health [5]. Based on the growing controversy regarding its definition, the European Society of Intensive Care Medicine convened the Third International Consensus Task Force to redefine the concept of sepsis [6]. The redefinition followed continuous deliberations among experts coupled with an increased review of the literature to find a more accurate framework. Ultimately, the consensus revised and validated a new concept of diagnosing sepsis called sepsis-3 [7].

The rarity of intensive care units across the world means that any obscurity in the definition of sepsis can undermine public health. In particular, the intensive care resources in China are limited based on its economic situation as a midincome developing country [8]. Besides, the unavailability of adequate resources within the healthcare sector undermines efforts of accurately managing sepsis. In this regard, a more accurate and straightforward strategy is necessary for facilitating the admission of severely ill patients in intensive care units [9, 10]. This paper follows the criticism of the sepsis-1 definition, which asserts the individuals' systemic inflammatory response syndrome to infection as primary in determining sepsis. In this initial definition, individuals would be diagnosed with sepsis upon fulfilling at least two SIRS criteria based on their inflammatory response. It is the lack of specificity in this definition that gave rise to new definitions in the form of sepsis-2 and sepsis-3 [11, 12].

Despite the emergence of new definitions, the first definition (sepsis-1) is more widely used across the world. In particular, the absence of validation of sepsis-3 means that most countries rely on previous definitions for admission of patients to intensive care units. In China, the primary diagnostic criteria have been based on infection and satisfaction of two SIRS criteria defined in sepsis-1 [13]. Consequently, it is necessary that sepsis-3 criteria are immediately validated to facilitate the precise diagnosis of sepsis. In the current study, the prognostic accuracy of SOFA and SIRS was compared by analyzing the traits of patients satisfying the first and third diagnostic criteria of sepsis-1 and sepsis-3, respectively. In achieving this objective, the research experiment derived data from the Medical Information Mart for Intensive Care-III (MIMIC-III) database.

The article "Evaluation of Sepsis-1 and Sepsis-3 Diagnostic Criteria in Patients with Sepsis in Intensive Care Unit" was published in 2023. Journal: J Healthc Eng.

## 2. Methodology

### 2.1. The Database

The analysis of patient information is based on data contained in the Medical Information Mart for Intensive Care-III (MIMIC-III) database. This database is freely accessible and was established by the Beth Israel Deaconess Medical Center (BIDMC) and MIT's Computational Physiology Laboratory. The database is a voluminous single-center database containing information pertaining to 38,000 adults who were admitted to the BIDMC in the 11 years leading up to 2012. The database contains de-identified information, thereby maintaining the confidentiality and privacy of patients. Furthermore, the database integrates vital sign measurement, laboratory results, diagnostic codes, medications, demographic data, and fluid balance entries [14, 15]. All this information was necessary for addressing the objectives of this research paper. It is freely and publicly accessible to researchers across the world and has medical information on 40,000 patients spanning slightly over a decade. In accessing the information, we had to undertake a training course on research handling of human subjects in research. Besides, we signed a data use agreement that mandated us with the responsibility of ethically handling the data and the mandatory adherence to collaborative research principles.

### 2.2. Study Design

The identification of patients with sepsis was conducted using the International Classification of Diseases (ICD-10-CM) diagnosis codes [16]. The data extraction from the records was limited to people of eighteen years and below, thereby excluding medical information on adults. The identification of both sepsis-1 and sepsis-3 patients was based on the fulfilment of the SIRS and SOFA criteria, respectively. Upon selecting this patient population, it will further be categorized into those who have a history of chronic organ disorder and those who do not have. The identification of patients with previous chronic organ disorders was based on a search from the database using the keywords. Using 28-day mortality as the benchmark outcome after admission to ICU, the study assessed the accuracy of SIRS and SOFA diagnostic criteria in predicting mortality within 28 days. The accuracy was ascertained using the area under the ROCs, receiver operator curves (ROCs), and specificity and sensitivity of the two criteria.

The article "Evaluation of Sepsis-1 and Sepsis-3 Diagnostic Criteria in Patients with Sepsis in Intensive Care Unit" was published in 2023. Journal: J Healthc Eng.

### 2.3. Derivation of Data

The derivation of the data from the MIMIC-III database was based on the latest version of the database. In achieving this endeavor, the researchers used SQL software to query and mine data from the database. The database provided access to the DIAGNOSES_ICD table, which provided details of patients as prescribed in the ICD-10-CM codes of diagnoses [17]. The process involved the extraction of adults above the age of 18 years from the list of infected patients and used as the research subjects. The database presented information in a de-identified form, thereby concealing personal information on the patients. The CHARTEVENTS, INPUTEVENTS, LABEVENTS, and OUTPUTEVENTS tables provided the primary variables for the SOFA and SIRS standards. These variables would then be extracted from the database for use in the research process. In an effort to include more septic patients, the querying of the data was based on an extended time window of between 12 hours preadmission and two days postadmission into the ICU. In the end, the researchers used the NOTEEVENTS table to extract PMH information related to the identified subjects, thus helping in categorizing patients who had previous organ dysfunctions.

### 2.4. Procedure and Diagnosis

The querying of participants in the study was based on suspected cases of infection and sepsis in patients. In particular, patients put on antibiotics within the first two days of admission and with cultures were suspected of having infections [18]. These data were retrieved from the database before further being grouped into two categories. The first category was based on sepsis-1 criteria as defined using the SIRS threshold. In this regard, the clinical criteria for this category of subjects were the evidence of suspected infection coupled with the satisfaction of SIRS criteria. The diagnosis of sepsis-1 is appropriate where patients satisfy two of the SIRS criteria. These components include temperature below 36^o^C or above 38^o^C; respiratory rate that exceeds 20 breaths per minute; heart rate exceeding 90 beats per minute; and leukocytes that exceed 12,000/*μ*L or below 4,000/*μ*L. Similarly, the procedure included querying for sepsis-3 in patients by identifying their SOFA scores in patients with suspected infections. Those with scores above two within two days of admission into the ICU were considered to satisfy the SOFA requirements.

The article "Evaluation of Sepsis-1 and Sepsis-3 Diagnostic Criteria in Patients with Sepsis in Intensive Care Unit" was published in 2023. Journal: J Healthc Eng.

#### 2.4.1. Statistical Analysis

The retrieved data were further analyzed using a combination of two softwares: SPSS and R software. Inherently, this software was appropriate for both management and analysis of retrieved data. As noted in Bryman and Cramer, the SPSS software is largely used in the quantitative analysis because of its potential to analyze and mine relevant data variables [19]. Similarly, the R software was useful in the research process because of its potential for exploration, modeling, and visualization of data. In particular, the chi-square test was significant in comparing the specificity, mortality, and sensitivity of the data. Indeed, chi-square tests are effective in examining the variances across categorical variables within the same population or data set [20]. In turn, the chi-square test was used in assessing the statistical significance of different variables and data. In contrast, the *Z* test was used to compare variables of the area under the curves (AUCs). Inherently, *Z* tests are effective in comparing multiple independent proportions by estimating the standard normal deviate in a population [21]. The level of statistical significance was capped at a probability value of less than 0.05.

## 3. Results

The process of screening the Medical Information Mart for Intensive Care-III (MIMIC-III) database resulted in the identification of 21,368 patients with infections from the hospital admissions in the database. In particular, only 46% of all admissions were identified as infected patients. Besides, the results also portray a significant variance in the number of survivors and nonsurvivors during the 28-day period after admission (see Table 1). The results of the study portray a higher mean age for survivors compared with nonsurvivors, with the former recording a mean age of 64.63 and a standard deviation of 16.86. In contrast, nonsurvivors had a younger age at a mean of 70.53 and a standard deviation of 14.54. Still, a significant majority of nonsurvivors and survivors were hospitalized using ambulances, thus indicating emergencies at the time of admission. Of all admissions, 86.45% of nonsurvivors and 93.64% of survivors were hospitalized through ambulances based on a significance level of 0.001.

The study further finds a higher risk of mortality among patients in intensive care facilities relative to others. Indeed, those in ICU had a probability of 64.32% succumbing to death compared with 48.62% in other patients with a significance level of less than 0.001. The findings of the study also indicate a marginal difference between the SOFA scores in survivors and nonsurvivors. While survivors had a score of 4.0 (2.0∼6.0), nonsurvivors had a significantly higher rate at 7.0 (4.0∼10.0) at a significance level of <0.001. Of the 21,368 infected patients derived from the database, 92.4% met the sepsis-1 criteria on their first day of admission by scoring at least two SIRS scores. In contrast, 86.3% of these infected patients were qualified for sepsis-3 based on a score of above two in the SOFA criteria. The results also indicate a significantly higher mortality rate within 28 days of admission in sepsis-3 patients compared with sepsis-1 (see Table 2). In particular, the significance levels for ICU mortality, final mortality, hospital mortality, and 28-day mortality were 0.006, 0.001, 0.006, and 0.013, respectively.

The article "Evaluation of Sepsis-1 and Sepsis-3 Diagnostic Criteria in Patients with Sepsis in Intensive Care Unit" was published in 2023. Journal: J Healthc Eng.

The subsequent improvement of the definition of sepsis and its diagnostic criteria was actualized based on multiple factors. In part, the SIRS criteria were not very effective in identifying sepsis among infected individuals [22]. As noted in the study by Fleischmann et al., about 12% of patients admitted into intensive care units did not meet the SIRS criteria for sepsis even though they had contracted the condition and had high mortality rates [23]. The older definition and diagnostic criteria of sepsis (sepsis-1) were not effective in identifying cases of sepsis among ICU patients. The results of this study have portrayed the need for modification of the older diagnostic criteria based on the variance between patients who met the sepsis-3 criteria and those who met the sepsis-1 criteria [24]. 6.87% of the patients who met the diagnostic criteria for sepsis-3 did not meet the criteria for sepsis-1, a finding that supports the modification of the old diagnostic criteria for sepsis. This means that the sepsis-1 criteria were not effective and did not accurately identify all the patients who had sepsis infections. Perhaps more worrying is that these patients had a mortality rate of 10.78% within 28 days after admission to intensive care units. The high mortality rate means that many patients risk death by not being diagnosed as having sepsis because of the inadequacies of traditional diagnostic criteria.

A smaller percentage of the sepsis-1 patients did not meet the SOFA criteria for sepsis-3. In particular, only 13.42% of sepsis-1 patients were termed as sepsis-1 specific patients and had a 28-day mortality rate of 7.05%. On the other hand, 6.87% of sepsis-3 patients were sepsis-3 specific patients because they did not meet the SIRS criteria. This group of patients had a 28-day mortality rate of 10.78% (see Table 3). Inherently, sepsis-3 specific patients had a significantly higher mortality rate compared with sepsis-1 specific patients. Sepsis-1 specific patients with no preexisting organ dysfunction had a significantly lower mortality rate of 6.39% compared with sepsis-3 specific patients without preexisting organ dysfunction, which was 9.11%. A similar trend was observed among sepsis-1 specific patients with preexisting organ dysfunction whose mortality rates were lower than sepsis-3 specific patients with preexisting conditions. Despite the variance, the difference was not statistically significant at a *p* value of 0.153.

The article "Evaluation of Sepsis-1 and Sepsis-3 Diagnostic Criteria in Patients with Sepsis in Intensive Care Unit" was published in 2023. Journal: J Healthc Eng.

The use of organ dysfunction within 24 hours postadmission as qualifying criteria in diagnosing sepsis in patients is also flawed. In particular, the reliance on this proposition, coupled with the assumption of the basal parameters before a patient's admission, fails to consider potential underlying diseases. The results of this study, therefore, indicate the possibility of some patients having severe sepsis and still having prior organ dysfunctions, which were not attributable to the sepsis infection. In addressing the identified challenge, the study grouped patients in the MIMIC-III database into categories based on known underlying conditions. When the underlying conditions were not considered, a significant number of sepsis-1 patients (18.31%) did not satisfy the sepsis-3 diagnostic criteria. Surprisingly, this set of patients had a 28-day mortality rate of 6.46%. In contrast, the exclusion of underlying conditions revealed that only 6% of sepsis-3 patients failed to meet the criteria for sepsis-1 with a mortality rate of 8.9% over the 28-day period. Based on these results, the more current diagnostic criteria (sepsis-3) were missed out on the diagnosis of sepsis patients compared with the traditional (sepsis-1) criteria [16]. The mortality rates over 28 days reveal that the specificity of sepsis-3 criteria was more than that of sepsis-1, with an inverse result observed in terms of the sensitivity. In this regard, the improvement to the sepsis-3 criteria is more beneficial based on its potential to correctly diagnose more sepsis patients [25]. Although the sepsis-1 criteria were effective in correctly diagnosing those who have no sepsis, diagnosing more patients who have sepsis accurately is more beneficial.

We then analyzed the clinical factors associated with the sepsis-1 and sepsis-3. The results are presented in Tables 4 and 5. As shown in the tables, the clinical factors associated with sepsis-1 and sepsis-3 were the same clinical factors. The age of the patients, the admission type to ICU, the APACHE II score, the SAPS, and the MPM were associated with the sepsis-1 and sepsis-3.

The article "Evaluation of Sepsis-1 and Sepsis-3 Diagnostic Criteria in Patients with Sepsis in Intensive Care Unit" was published in 2023. Journal: J Healthc Eng.

## 4. Discussion

The results of the study portray a significant challenge in the use of the SOFA diagnostic criteria for sepsis-3. In particular, the determination of the onset of organ dysfunction is not attainable, thus imparting doubts on whether the dysfunction occurred before or after the onset of the infection [25]. In scenarios where organ dysfunction is proven by health records, its severity before the infection is not easily determined [10]. Moreover, most of the health records in developing countries, including China, are not very accurate or well established, thus compounding the revelation of time of organ dysfunction [10]. Even in some developed countries, it becomes challenging to retrieve detailed information on the functioning of organs in patients. As noted in the diagnostic criteria for sepsis-3, a patient must achieve a score of at least 2 [24, 26, 27]. However, determining the effect of an infection on the organ dysfunction is highly challenging. Even though this problem was addressed in the proposition of the assumption of the baseline SOFA score to be zero, this proposition is not accurate. Indeed, this proposition may contribute to instances of patients with flu being misdiagnosed as having sepsis based on the assumption of basal parameters of the patient before their admission [28].

The onset of sepsis in patients impairs the ability of the host to regulate their response to the infection. In particular, the pathophysiological problem may result in potential death or heightened organ dysfunction [9]. The continued presence of sepsis in patients increases the risk of death based on a continuum of diseases. The sepsis-1 diagnostic criterion has limited specificity because of the absence of exclusivity in associating the requisite conditions to infection. That notwithstanding, the SIRS criterion is broad in its scope, thus increasing its sensitivity and accuracy in identifying sepsis in patients. In clinical practice, it would be fatal to wait until the manifestation of life-threatening organ dysfunction for diagnosis of sepsis to be made. Despite its criticism, therefore, the sepsis-1 criterion was based on the need to make early and almost instant identification of sepsis in patients [23]. Through high rates of disease identification in patients, physicians and other healthcare professionals would help provide requisite interventions, thus reducing the potential for high mortality rates among sepsis patients [29].

## 5. Conclusion

The results of the study confirm the need for improvements on the traditional diagnostic criteria for sepsis infection. In particular, the use of the sepsis-3 diagnostic criteria is more specific and narrow than that of the sepsis-1 criteria. A shift to the SOFA diagnostic criteria (sepsis-3) can significantly improve the specificity of identifying cases of sepsis to guide admission to critical care units. On the other hand, the narrow diagnostic criteria in sepsis-3 may contribute to higher misdiagnosis cases, thus delaying treatment for patients with sepsis. Besides, the primary goal of accurately defining sepsis is to enable early identification and effective treatment interventions. Based on the limitations of each of the two diagnostic criteria, it is important to consider their associated specificity and sensitivity rates when applied to ICU patients. Consequently, there is an inherent need to consider the broader spectrum of sepsis and risks stratification in choosing accurate diagnostic criteria.

The article "Evaluation of Sepsis-1 and Sepsis-3 Diagnostic Criteria in Patients with Sepsis in Intensive Care Unit" was published in 2023. Journal: J Healthc Eng.

## Figures and Tables

**Table 1:** Clinical comparisons of survivors and nonsurvivors in 28 days.

Variables	Overall (*n* = 21368)	Survivors (*n* = 16456)	Nonsurvivors (*n* = 4912)	*p* value
Age (mean + SD)	65.71 + 15.34	64.63 + 16.86	70.53 + 14.54	<0.001
Gender				<0.001
Male, *n* (%)	11169 (52.27)	8417 (51.15)	2669 (54.34)	
Female, *n* (%)	10199 (47.73)	8039 (48.85)	2243 (45.66)	
Admission type				<0.001
Elective, *n* (%)	1241 (5.81)	1228 (7.46)	205 (4.17)	
Emergency, *n* (%)	19497 (91.24)	14636 (88.94)	4561 (92.86)	
Urgent, *n* (%)	630 (2.95)	592 (3.60)	146 (2.97)	
Care unit				<0.001
MICU, *n* (%)	11312 (52.94)	8468 (51.46)	3013 (61.34)	
SICU, *n* (%)	3308 (15.48)	2608 (15.85)	650 (13.24)	
CCU, *n* (%)	2791 (13.06)	2080 (12.64)	616 (12.54)	
CSRU, *n* (%)	2038 (9.54)	1827 (11.10)	277 (5.64)	
TSICU, *n* (%)	1919 (8.98)	1473 (8.95)	356 (7.24)	
SIRS, median (IQR)	3.0 (2.0∼4.0)	3.0 (2.0∼4.0)	3.0 (3.0∼4.0)	<0.001
SOFA, median (IQR)	4.0 (2.0∼7.0)	4.0 (2.0∼6.0)	7.0 (4.0∼10.0)	<0.001

**Table 2:** Mortality rate comparisons for sepsis-1 and sepsis-3 criteria.

Criteria	28-day mortality	ICU mortality	Hospital mortality	Final mortality
Sepsis-1 (infection plus SIRS>2)	16.44%	17.12%	17.12%	54.64%
Sepsis-3 (infection plus SOFA>2)	17.46%	18.32%	18.41%	59.80%
*p* value	0.013	0.006	0.006	0.001

**Table 3:** AUCs of mortality prediction for different patient groups.

Group	AUC for SIRS (95% CI)	AUC for SOFA (95% CI)	*p* value
1	0.587 (0.583∼0.610)	0.714 (0.703∼0.724)	<0.001
2	0.584 (0.573∼0.599)	0.698 (0.646∼0.712)	<0.001
3	0.607 (0.591∼0.623)	0.702 (0.689∼0.718)	<0.001

**Table 4:** Factors associated with the sepsis-1.

Clinical parameters	Odds ratio	95% CI	*p* value
Age			0.026
≤60	Reference		
>60	2.13	1.56–3.46	
Gender			0.125
Male	Reference		
Female	1.23	0.87–1.56	
Admission type			0.013
Elective	Reference		
Emergency	1.57	1.33–2.16	
APACHE II	1.95	1.49–2.36	0.002
SAPS	1.88	1.62–2.03	0.006
MPM	1.57	1.33–1.92	0.004

The article "Evaluation of Sepsis-1 and Sepsis-3 Diagnostic Criteria in Patients with Sepsis in Intensive Care Unit" was published in 2023. Journal: J Healthc Eng.

**Table 5:** Factors associated with the sepsis-3.

Clinical parameters	Odds ratio	95% CI	*p* value
Age			0.017
≤60	Reference		
>60	2.18	1.57–3.88	
Gender			0.236
Male	Reference		
Female	1.56	0.87–2.11	
Admission type			0.011
Elective	Reference		
Emergency	1.77	1.38–2.26	
APACHE II	1.88	1.79–2.15	0.001
SAPS	1.45	1.33–1.79	0.014
MPM	1.57	1.13–1.84	0.001

## Data Availability

The simulation experiment data used to support the findings of this study are available from the corresponding author upon request.
